The article "Application of edge computing and GIS in ecological water requirement prediction and optimal allocation of water resources in irrigation area" was retracted in 2024. Reasons: false authorship; unreliable results or conclusions; concerns about the peer review.

# Application of edge computing and GIS in ecological water requirement prediction and optimal allocation of water resources in irrigation area

**DOI:** 10.1371/journal.pone.0254547

**Published:** 2021-07-29

**Authors:** Yang Li, Jiancang Xie, Rengui Jiang, Dongfei Yan

**Affiliations:** State Key Laboratory of Eco-hydraulics in Northwest Arid Region, Xi’an University of Technology, Xi’an, 710048, China; Ministry of Natural Resources North Sea Bureau, CHINA

## Abstract

The purposes are to use water resources efficiently and ensure the sustainable development of social water resources. The edge computing technology and GIS (Geographic Information Science) image data are combined from the perspective of sustainable development. A prediction model for the water resources in the irrigation area is constructed. With the goal of maximizing comprehensive benefits, the optimal allocation of water quality and quantity of water resources is determined. Finally, the actual effect of the model is verified through specific instance data in a province. Results demonstrate that the proposed irrigation area ecological prediction model based on edge computing and GIS images can provide better performance than other state of the art models on water resources prediction. Specifically, the accuracy can remain above 90%. The proposed model for ecological water demand prediction in the irrigation area and optimal allocation of water resources is based on the principle of quality water supply. The optimal allocation of water resources reveals the sustainable development ideas and the requirements of the optimal allocation model, which is very reasonable. The improvement of the system is effective and feasible, and the optimal allocation results are reasonable. This allocation model aims at the water quality and quantity conditions, water conservancy project conditions, and specific water demand requirements in the study area. The calculation results have great practicability and a strong guiding significance for the sustainable utilization and management of the irrigation area.

## Introduction

As the social economy develops and the population increases rapidly, the world faces three major challenges: population, environment, and resources; especially, water resource has become one of the key issues [1]. Water resources are the material basis for human survival and social and economic development, an irreplaceable important natural resource and strategic economic resource, and an important guarantee for sustainable development [2]. The problem of water resources is global. However, the shortage of water resources and the worsening of water pollution are becoming increasingly serious today. A sharp contradiction between the supply and demand of water resources is formed, which is one of the most important factors restricting the current social and economic development [3]. At the same time, human health and the ecological environment system are seriously threatened. Since the 20th century, the emergence of water shortages all over the world has led to the struggle for the right to control water resources. In the next century, it will likely trigger hostility between many countries and races [4]. Therefore, how to scientifically develop, utilize, and protect water resources, realize the sustainable development of ecological environment and social economy, and maximize the economic, environmental, and social benefits of water resources is a problem that needs to be solved urgently all over the world [5]. To realize the sustainable use of water resources and ensure the sustainable development of society, economy, and environment, as the most important means to solve water resources, research on the optimal allocation of water resources has important theoretical significance and practical value.

The main approaches to solving the contradiction between water supply and demand are increasing revenue, reducing expenditure, controlling pollution, and managing water resources. Increasing revenue means that for areas with abundant water resources and low water resources development and utilization, investment can be increased, water conservancy projects and facilities can be built, and new water sources can be developed to improve the efficiency of water use in the area and increase water supply capacity [6,7]. Reducing expenditure refers to that at areas with relatively poor water resources and high utilization of water resources, management measures can be taken to increase people’s awareness of water conservation, and water-saving technologies and methods can be adopted to reduce water waste and establish a water-saving society. It is a long-term strategy to alleviate the contradiction between water supply and demand and realize the sustainable use of water resources [8]. Controlling pollution refers to that at areas with severe water pollution, the wastewater utilization rate, the discharge rate of production and domestic sewage, and current water quality can be improved by strengthening environmental awareness, increasing water pollution control efforts, building sewage treatment equipment, improving [9]. Managing water resources refers to the organization, coordination, supervision, and dispatch of water resources development and utilization. The optimal allocation of water resources is one of the core contents of water management. It uses systematic analysis methods to comprehensively plan the amount of water resources in water-deficient areas, and apply scientific methods to change the traditional management models [10]. The allocation of limited water resources can be optimized according to the importance of the production sector and the size of the benefits, thereby changing the traditional management models and methods and optimizing the allocation of limited water resources. In this regard, the water resources can be utilized comprehensively and efficiently, and sustainable social and economic development can be ensured.

The innovative points are: (1) the correlation between water resources and the ecological environment is clarified, the ecological water demand is adequately divided, and relevant calculation methods are provided. (2) The MEC (Multi-access Edge Computing) method is applied to predict the ecological water demand in the irrigation area, helping urban water resources connect to the Internet of Things for urban development, as well as improving the utilization rate of water resources. (3) GIS is combined with multiple methods to optimize the design and allocate the relevant allocation plans, which can greatly promote the practical application of urban water resources.

## Literature review

### Irrigation area ecosystem

Irrigation areas are important to China’s agricultural large-scale production and the bases of commodity grain, cotton, and oil. They are the vital infrastructure for China’s agricultural, rural, and even national economic development. Irrigation area ecosystem refers to the ecological functional unit of material circulation, energy flow, and information transmission between various living organisms and non-biological environments based on agricultural organisms within the spatial scope of the agricultural irrigation area, with the active participation of human beings through water and soil engineering and other measures [11]. Arcari et al. (2019) demonstrated the feasibility of applying the dynamic programming method to the optimal water allocation in the irrigation season and established a corresponding deterministic dynamic programming model [12]. Ricart et al. (2020) took the California Empire River Valley farm as the research object. They proposed the optimal water demand plan for the farm according to different irrigation volumes and water quality. They also used linear programming to maximize the benefits of waterman resources to obtain the optimal planting structure [13]. Wang et al. (2021) conducted a lot of research on the optimal allocation of irrigation water during the crop growing season to obtain the maximum economic benefits using stochastic control principles and methods [14]. Liu et al. (2021) proposed a daily real-time optimal scheduling model combining simulation and DP (Drucker-Prager). They considered the multi-functionality of water and the relationship between multiple interests, emphasized the cooperation between decision-makers and decision analysts, and established a multi-level model of water resource allocation, which reflected the multi-objective and hierarchical structure of water resources allocation [15]. Chien et al. (2021) used dynamic programming to solve the optimal irrigation strategy for water shortage irrigation based on the dynamic water production function model. Combining the crop growth model and stochastic dynamic programming with 2D state variables, they studied the seasonal irrigation water allocation in the irrigation area [16].

### Theory of ecological water demand

Ecological water demand refers to water used to improve water quality, coordinate ecology, and beautify the environment. It is not just a biological water demand and water consumption, but a systematic ecological concept [17]. Many scholars have researched the theory of ecological water demand. Yi et al. (2018) studied ecological water demand around the amount of water required to maintain the balance of the ecosystem, ecological restoration, and vegetation growth and survival in different regions. They pointed out the various states of ecological water demand. In fact, this ecological water demand referred to the ecological water demand of vegetation in this arid area environment [18]. Similarly, the definition of vegetation ecological water demand is very different given different research objects and points of view. Zhang et al. (2019) believed that vegetation ecological water demand referred to the amount of water consumed to maintain the stability of the vegetation ecosystem at a specific scale and environmental state [19]. Yamamura et al. (2021) believed that vegetation ecological water demand was the amount of water consumed to maintain the stability of the ecosystem, ecological protection, and ecological construction based on the characteristics of the ecological environment in the arid area of northwestern China. Results demonstrated that given the obvious differences in the environmental characteristics of different regions, the focus of vegetation ecological water demand would also be different, and its calculation method had significant regional characteristics and generally lacked the support of long-term data, which was uncertain in guiding the optimal allocation of water resources [20]. Yuan et al. (2021) pointed out that according to the different climate environment, hydrogeology, and vegetation types, the calculation methods of vegetation ecological water demand were also different. At present, common research methods included the area quota method, the phreatic evaporation method, the vegetation ecological water demand based on vegetation evapotranspiration, and the systematic research methods based on remote sensing and geographic information. They also clarified the advantages, disadvantages, and application ranges of various research methods in different regions [21].

### Review of recent works

Research on the irrigation area ecosystem has gradually tended to intelligent monitoring, focusing on providing different agricultural irrigation schemes. However, there is less research on water resource monitoring in the irrigation area ecosystem. Most research on ecological water demand emphasizes establishing the relationship between water resources and land use. Nevertheless, few studies on the actual ecological water demand prediction have been reported. Although many methods have been adopted to optimize the water resources, there is no significant improvement over the utilization rate of water resources. Therefore, in the present work, edge computing and GIS (Geographic Information Science) image data are combined to build an irrigation area water resource prediction model from the perspective of sustainable development. Afterward, an optimal allocation scheme for the quality and quantity of water resources is determined to maximize the comprehensive benefits. Eventually, the actual effect of the model is verified through specific province instance data. The research results have important reference value for promoting the green, healthy, and sustainable development of irrigation areas.

## Research methodology

### Optimal allocation of water resources

As per the decomposition and coordination technology of GIS system theory, the model coordination method is adopted to establish a model for the reasonable allocation of regional water resources and water volume [22,23]. There are three coordination layers in the optimization model of water volume. The first layer is based on the crop water production function, which solves the dynamic programming model for optimizing the irrigation system under the condition of insufficient irrigation for a single crop. Its role is to optimally allocate the irrigation water *X*_*k*_ and *Y*_*k*_ allocated to the *k*-th crop by the second layer during the crop’s growth stage, obtain the maximum benefit of the subsystem, and feed it back to the second layer. The second layer is a linear algorithm model that solves the optimal water allocation among multiple crops. Its role is to allocate the irrigation water volume *V*_*3*_ allocated to agricultural water by the third layer, perform optimal allocation among various crops in the irrigation area, pass the allocation plan to the first layer, accept the information feedback from the first layer for coordination and optimization, and transfer the information to the third layer after reaching its optimal. The third layer is the overall coordination layer, which is an edge computing algorithm model for solving the irrigation area’s water allocation optimization among various water-using departments. First, the initial value of the water consumption of each water-using department is preset and passed to the second layer. Then, it receives the information about coordination and optimization sent by the second layer to maximize the comprehensive benefit of the total system. After decomposition and coordination of optimization at all levels, the optimal irrigation system for various crops can be obtained, and the optimal water distribution process for the irrigation area can also be obtained. The above model divides the entire irrigation area into four water-using departments: industry, agriculture, ecological environment, and living. The allocation of agricultural water is divided into K subsystems according to the types of crops. Thus, the dimensionality of the problem is reduced through decomposition and coordination, making it easy to solve. The structure of the decomposition and coordination model of optimal water resource allocation in the irrigation area is displayed in Fig 1 below.

**Fig 1:** The optimal allocation plan of the water resource and water volume.

GIS adopts the mainstream GIS platform, advanced spatial data service, and scalable network map service, which can store, manage, and use spatial data in DBMS, widely release GIS maps, data, and metadata to network users, and support the construction of distributed, multi-tiered GIS applications. All geographic information is stored in the server or database. The electronic map layer data of the system can be centrally stored and maintained at different levels. A unified GIS server is established to store the electronic map layer database centrally. The layer data of all servers shall be based on the data of the GIS server, and the layer data of the GIS server shall be kept updated in real-time. The GIS data of each server of the system shall be kept consistent. It can be closely integrated with the database-based form file system to flexibly realize the mutual access of pictures, texts, and data. The system should have a strong drawing function, easily draw and output standard working drawings, support seamless overlay of multiple scale maps and image data processing functions, and directly overlay various image maps after coordinate correction. It can be well combined with popular relational databases, support spatial data storage of relational databases, meet the needs of digital map storage and application, and handle large amounts of data; its running speed also meets actual needs. The system should also provide a complete, convenient, and practical means of storing, querying, updating, and upgrading map data. To ensure the versatility of GIS and the reliability of maintenance and upgrades, geographic information systems should directly use vectorized electronic maps in common formats without any format conversion.

### Water resources allocation plan

The water quality and sources required by various water-using departments in the irrigation area are not the same. The four water-using departments of industry, agriculture, ecological environment, and living put forward different water quality requirements. The water quality requirements of various water-using departments are divided into three levels: I, II, and III. The water quality requirements on water used for living are the highest, which is Level I; the requirements on industrial water rank the second, which is Level II; the requirements on both agricultural and ecological water are Level III. The supply relationship between water resources and water-using departments follows the following principles of water quality: low-quality water cannot be supplied to high-level water-using departments, while high-quality water can be supplied to low-level water-using departments. High-quality water should be supplied to high-level water-using departments in prior; surpluses can be supplied to lower-level water-using departments [24]. Assuming that the water consumption of various water-using departments is *d*_*j*_ *(j = l*, *2*, *3*, *4)*, and the total amount of the three types of water that can be supplied by local water resources and external water resources are *Q*_*1*_, *Q*_*2*_, and *Q*_*3*_ [25], respectively, then:

$$d_{j}=Q_{1}+Q_{2}+Q_{3}$$ (1)

In (1), *d*_*j*_ refers to the water consumption of the *j*-th department, and *Q*_*1*_, *Q*_*2*_, and *Q*_*3*_ are the water consumption of the three different types of water provided to the *j*-th department. The specific optimal allocation plan of the water resources is illustrated in Fig 2.

**Fig 2:** Water resource allocation plan.

### GIS-based resource monitoring

Remote sensing monitoring is a technical means that uses remote sensing technology for monitoring, such as ground coverage, atmosphere, ocean, and near-surface conditions. Remote sensing monitoring collects electromagnetic wave information of the environment via aviation or satellites to monitor and identify environmental quality conditions far from environmental targets. It is an advanced environmental information acquisition technology that can quickly and comprehensively obtain large-area synchronous and dynamic environmental information, which is unmatched by other approaches. Therefore, it has been widely accepted, such as atmospheric and water quality remote sensing monitoring, marine oil pollution accident investigation, urban thermal environment and water thermal pollution investigation, urban green space, landscape and environmental background investigation, and ecological environment investigation and monitoring. GIS technology can effectively combine geographic graphic data with various information of traffic management to display more intuitively in space. Using GIS spatial analysis technology can efficiently assist transportation route planning, design, and decision-making. Using the data storage function of GIS technology can manage, inquire, analyze, count, and output the traffic data. Therefore, remote sensing and GIS are used for modeling in the present work.

At present, the latest research method is based on the regional differentiation law of vegetation growth water demand, which calculates the ecological water demand through the combination of GIS software and measured data. First, remote sensing and GIS technology are employed for spatial ecological zoning. Then the area of ecological zoning at all levels of the basin and the type of water demand are determined through the overlay analysis of ecological zoning and water resource zoning. Third, the spatial correspondence between ecological zoning and water resource zoning is analyzed to determine the scope and standard of ecological water consumption. The precipitation balance and water resource balance are analyzed with the basin as a unit, and the vegetation ecological water demand is calculated on this basis. This method is suitable for calculating the ecological water demand of vegetation in a large area, which has the characteristics of a large workload and complex technology [26]. The specific implementation process is shown in Fig 3.

**Fig 3:** GIS-based water resource monitoring.

### Edge computing processing

Edge computing uses the open platform that integrates network, computing, storage, and application core capabilities on the side close to the source of things or data to provide services nearby. Its applications are initiated on edges to generate faster network service response and meet the basic needs of the industry in real-time business, application intelligence, security, and privacy protection. Cloud computing can still access the historical data of edge computing. Edge computing can be completed in large-scale computing equipment, as well as small and medium-sized computing equipment and local networks. Devices used for edge computing can be mobile devices such as smartphones, PC (Personal Computer), smart homes, driverless cars, and other home terminals, or ATMs (Automatic Teller Machines), cameras, traffic lights, motors, pumps, power generators, or other sensors and other terminals. Edge computing emerges with the development of the Internet of Things (IoT). Regarding IoT, breakthroughs in edge computing mean that data analysis and control can be achieved through local devices without cloud processing. It will greatly improve the efficiency of data processing, reduce the cloud load, and provide users with a faster response.

Edge computing can utilize the wireless access network to provide nearby IT (Information Technology) services and cloud computing functions required by telecom users, creating a carrier-grade service environment with high performance, low latency, and high bandwidth, allowing consumers to enjoy uninterrupted high-quality network experience [27]. Because the prediction of ecological water demand in the irrigation area ecosystem is often delayed by the network, the data cannot be uploaded and processed quickly, so that the implementation of government policies often faces huge delays. MEC has the advantages of distributed computing, making it very suitable for dealing with the problems caused by water sensors. The sharpness of the edge is determined by the gradient of the image gray. The gradient is a vector, and *∇f* points out the fastest direction and amount of change in grayscale [28].

$$\nabla f=(\frac{\partial f}{\partial x},\frac{\partial f}{\partial y})$$ (2)

In (2), ∂*f*, ∂*x*, and ∂*y* are the numerical derivatives of *f*, *x*, and *y*. The gradient size is calculated as follows:

$$\left\|\nabla f\right\|=\sqrt{{\left(\frac{\partial f}{\partial x}\right)}^{2}+{\left(\frac{\partial f}{\partial y}\right)}^{2}}$$ (3)

The gradient direction is calculated as follows:

θ=(∂f∂y∂f∂x) (4)

The simplest edge detection operator is to approximate the gradient operator with the vertical and horizontal difference of the image:

∇f=(f(x,y)−f(x−1,y),f(x,y)−f(x,y−1)) (5)

The easiest way to look for edges is to calculate the vector for each pixel and then find its absolute value. According to this idea, the Roberts operator can be obtained:

g(x,y)={[f(x,y)−f(x+1,y+1)]2+[f(x,y+1)−f(x+1,y)]2}12 (6)

The Prewitt edge detection operator uses two directed operators (one horizontal and one vertical, generally called a template), each of which approximates a partial derivative:

$$p_{v}=\left(\begin{array}{ccc} -1 & -1 & -1\\ 0 & 0 & 0\\ 1 & 1 & 1 \end{array}\right)$$ (7)

$$p_{h}=\left(\begin{array}{ccc} 1 & 0 & -1\\ 1 & 0 & -1\\ 1 & 0 & -1 \end{array}\right)$$ (8)

In (8), *p*_*v*_ and *p*_*h*_ are the results of the horizontal and vertical operators. If the Prewitt operator is adopted to detect the edges of the data, the horizontal and the vertical operators can be used first to convolve the image, and two matrices will be obtained. Without considering the boundary, M1 and M2 are the same sizes as the original image, and they respectively represent the two partial derivatives at the same position in the image M. The two numbers corresponding to the positions of M1 and M2 are squared and added to obtain a new matrix **G**, where **G** represents the gradient value of each pixel in **M** (an approximation). Then the edge image can be obtained through threshold processing. Assuming that the gray level of the image satisfies the following relationship:

$$M_{x,y}=\alpha x+\beta y+\gamma$$ (9)

In (9), α and β are gradient coefficients, and *γ* is the correlation coefficient. Obviously, the pixel value in the 3×3 neighborhood of the current pixel is:

$$\left(\begin{array}{ccc} -\alpha -\beta +\gamma & -\alpha +\gamma & -\alpha +\beta +\gamma \\ -\beta +\gamma & \gamma & \beta +\gamma \\ \alpha -\beta +\gamma & \alpha +\gamma & \alpha +\beta +\gamma \end{array}\right)$$ (10)

The vertical and horizontal operators are defined as follows:

$$\left(\begin{array}{ccc} -a & -b & -a\\ 0 & 0 & 0\\ a & b & a \end{array}\right)$$ (11)

$$\left(\begin{array}{ccc} -a & 0 & a\\ -b & 0 & b\\ -a & 0 & a \end{array}\right)$$ (12)

In (12), *a* and *b* are the pixel values in the horizontal and vertical directions, respectively. These two templates are employed to convolve the current pixel, and the directional derivative obtained is:

$$\begin{array}{l} g_{x}=2\beta (2a+b)\\ g_{y}=2\alpha (2a+b) \end{array}$$ (13)

The gradient size at the current pixel is:

$$G=2(2a+b)\sqrt{\alpha^{2}+\beta^{2}}$$ (14)

Obviously:

2(2a+b)=1 (15)

The template obtained by taking *a = b* = 1/6 is 1/6 times the Prewitt operator. The detailed algorithm flow is shown in Fig 4.

**Fig 4:** Flowchart of MEC processing.

Based on the principle of energy balance, soil moisture and farmland evapotranspiration are considered to monitor drought conditions in real-time. It makes full use of modern remote sensing technology. Some of the physical quantities are retrieved from remote sensing images. Some of the daily and ten-day meteorological data from the Meteorological Bureau and the ground-measured data need to be combined with the topographic map of the study area under the support of GIS. The CWSI is calculated point by point according to the resolution of the remote sensing image, and the final calculation result is superimposed with the topographic map to obtain the required drought distribution map and other forms of results. Hence, the crop water shortage model can be complicated, involving the integrated processing of images, graphics, and data. Its calculation accuracy is related to the true degree of drought monitoring, and the calculation speed is associated with whether the drought can be monitored in real-time [29].

## Results and discussions

### Model performance analysis

Fig 5A–5D show the predictions of annual water demand at the planning level, each level of water resources at the planned level under Level I water resources, the water resources at Level II, and the water resources status at Level III. Under the annual guarantee rates, the water volume of the irrigation area I and II can meet the requirements of living water and industrial water. When P = 50%, the total water supply of the irrigation area in 2009 was slightly larger than the total water demand, and the total water supply of irrigation area water resources in 2019 was less than the total water demand. When P = 75% and P = 95%, the total water supply volume of the irrigation area in 2009 and 2019 could not meet the total water demand. Thus, there is no shortage of water quality in the irrigation area; instead, the total water is in shortage, which requires optimizing the allocation of water resources in the irrigation area.

**Fig 5:** Water resources status of planning levels under different year parameters.

As shown in Tables 1 and 2, the proposed model is compared with those in the latest literature [30]. As the number of different images increases, the accuracy of the model continues to improve. Regarding model performance, the proposed ecological water demand prediction model based on mobile edge computing and GIS performs better than the prediction model. In the literature [31], due to the CNN utilized, the processing time of the model is better; however, for agricultural production, the issue of cost needs to be considered. Therefore, the proposed model is relatively more suitable for practical analysis.

**Table 1:** Accuracy comparison of different models.

Accuary (%)	The proposed model	Literature [30]	Literature [31]	Literature [32]
0	0.8664	0.7745	0.8247	0.6925
50	0.8929	0.7248	0.8036	0.6543
100	0.9031	0.7345	0.8429	0.6825
150	0.9123	0.7689	0.8543	0.6943
200	0.9224	0.7796	0.8686	0.7077
250	0.9256	0.7815	0.8742	0.7125
300	0.9313	0.7912	0.8947	0.7215
350	0.9416	0.8014	0.8996	0.7313

**Table 2:** Running time comparison of different models.

Time (s)	The proposed model	Literature [30]	Literature [31]	Literature [32]
0	23	96	20	236
50	30	106	28	249
100	36	117	35	286
150	42	128	40	295
200	50	186	49	306
250	62	193	60	378
300	70	206	68	398
350	74	253	70	409

### Optimal allocation results of water resources

Fig 6A–6F respectively present the water resource allocation results of the water demand volume, surface runoff, groundwater, and crossing rivers when P = 50%, P = 75%, and P = 95% in 2009 and P = 50%, P = 75%, and P = 95% in 2019. Fig 7A–7F respectively show the water resource allocation results of irrigation water, total water supply, water shortage, and supply-demand ratio when P = 50%, P = 75%, and P = 95% in 2009 and P = 50%, P = 75%, and P = 95% in 2019. Compared with the situation in 2009, the irrigation area has slightly reduced water demand due to the adjustment of the planting structure in 2019. However, with population growth and social and economic development, the irrigation area has increased water consumption for industry, living, and ecological environment. Therefore, the total water demand of the irrigation area is increasing. When P = 75%, the water demand of the irrigation area in 2009 reached 276.1 million m^3^. In 2019, the water demand of the irrigation area increased to 284.7 million m^3^. However, the water resource of the irrigation area comes from crossing rivers, and there are no large water storage projects in the irrigation area; the water supply of the irrigation area’s water resource has become less able to meet the requirements of water demand under the condition of water intake restrictions from the crossing rivers. When P = 75%, the water shortage of the irrigation area in 2009 reached 57.03 million m^3^ and increased to 65.9 million m^3^ in 2019; meanwhile, the supply-demand ratio dropped from 79.3% in 2009 to 76.9% in 2019. Therefore, the irrigation area should increase the water withdrawal capacity of the crossing rivers and build water storage projects to store water in the season when it is less demanded, thereby alleviating the water pressure during the peak water consumption seasons.

**Fig 6:** Water resource allocation results of the water demand volume, surface runoff, groundwater, and crossing rivers.

**Fig 7:** Water resource allocation results of irrigation water, total water supply, water shortage, and supply-demand ratio.

### Benefit analysis of water resources

Fig 8A–8F respectively present the water resource allocation results of different crops, stages, and years when P = 50%, P = 75%, and P = 95% in 2009 and P = 50%, P = 75%, and P = 95% in 2019. Due to the high comprehensive benefits, the water supply of living water can reach the maximum demand under all levels and guarantee rates. The living water consumption in 2009 was 6.65 million m^3^ and 10.27 million m^3^ in 2019. However, the comprehensive benefits of industrial water are low, and only the minimum water demand requirement can be guaranteed in the case of water shortage. When P = 50%, the industrial water consumption in 2009 was 5.96 million m^3^; when P = 75% and P = 95%, due to water shortage, the industrial water consumption in 2009 was only 5.4 million m^3^. In 2019, the water consumption was 8.64 million m^3^ under all guarantee rates. Agriculture and the ecological environment are the two principal water-using departments in the irrigation area, which are also the two departments with serious water shortages. Agriculture has the most serious water shortage due to the low efficiency of agricultural water use; the coefficient of irrigation water utilization is only 0.44, indicating an extremely serious waste. Analysis suggests that if the irrigation water utilization coefficient reaches 0.7, the irrigation area guarantee rate will reach at least 75%. Therefore, it is necessary to vigorously transform the irrigation area canal system to improve water efficiency.

**Fig 8:** Water resource allocation results of different crops, stages, and years.

Fig 9A–9F show the benefit analysis of water resource allocation for different crops, stages, and years when P = 50%, P = 75%, and P = 95% in 2009 and P = 50%, P = 75%, and P = 95% in 2019. 2Compared with 2009, the agricultural water shortage in 019 was more serious; however, due to the adjustment of the agricultural structure, the planting area of cash crops increased from 80,000 hm^2^ in 2009 to 10,000 hm^2^, and the agricultural benefit was slightly improved than that in 2009. When P = 75%, the agricultural output value in 2009 was 51.89 million yuan; in 2019, it increased to 506.65 million yuan. It shows that the development of cash crops is an effective means to increase agricultural income while ensuring the output of important crops. When water distribution is performed between crops, the water guarantee for crops with higher economic output efficiency is better than that of crops with lower economic output efficiency. Besides, in each growth stage of a crop, water guarantees at critical growth stages should be provided rather than non-critical stages to efficiently use the water resources. Thus, the irrigation system obtained from the model is reasonable.

**Fig 9:** Benefit analysis of water resource allocation for different crops, stages, and years.

## Conclusions

From the perspective of sustainable development, an ecological water demand prediction model is constructed combining edge computing and GIS technology based on the comprehensive analysis of the current research on the optimal allocation of water resources. This model collects image data using GIS technology and divides different water resources timely and rapidly using edge computing data processing, thereby clarifying the relationship between water resources and the ecological environment. According to the corresponding results, an optimal allocation scheme for water resources is designed. This scheme aims at maximizing comprehensive income. Moreover, the effectiveness of the proposed model is proved through specific examples. Although the corresponding water prediction model and water resource optimization scheme have been constructed, there are several shortcomings in the present work. First, edge computing is highly dependent on local data and calculators, so that the algorithm processing efficiency and time are obviously weaker than other models. Second, although edge computing and GIS technology are used, many works have also used deep learning and neural networks for model optimization. These two aspects will be the research focuses in the future, in an effort to build a comprehensive urban water resource IoT system, construct a suitable water resource optimal allocation model, and realize the sustainable use of water resources.

## Supporting information

S1 Data (ZIP)
